# Related Factors and Economic Burden Evaluation of Nosocomial Infection in Patients with Chronic Kidney Disease

**DOI:** 10.1155/2022/9889917

**Published:** 2022-08-24

**Authors:** Jinxian Wang, Ling Zhang, Zhaoxia Yang, Ju Liu, Wei Guo

**Affiliations:** ^1^School of Public Health, Capital Medical University, Beijing, China; ^2^Hospital Infection Control Division, Shijingshan Teaching Hospital of Capital Medical University, Beijing Shijingshan Hospital, Beijing, China

## Abstract

Kidney disease in China has the characteristics of “three highs and one low“, namely high incidence, high disability rate, high treatment cost and low awareness. The main outcome is a progressive deterioration of renal function that is not easily corrected, and patients are often hospitalized repeatedly due to factors such as infection, fatigue, lack of medication, water and electrolyte imbalances. It not only accelerates the deterioration of renal function, but also easily causes psychological problems and seriously affects the quality of life of patients. Kidney is an organ with dual functions of endocrine and material metabolism in the human body, and plays an important role in both physiological and pathological processes. Its main functions include urine generation, renal tubular reabsorption, regulation of water and electrolyte metabolism, and endocrine functions. Chronic kidney disease is defined by an unexplained decrease in GFR over three months. At present, clinicians usually take drug corrective measures only when CKD patients have intermediate and advanced PEM with abnormal index examinations (such as decreased plasma albumin, anemia, etc.), and the clinical efficacy is not stable. At present, there are few studies on the related factors and economic burden of nosocomial infection in patients with chronic kidney disease. This study understands the nutrient intake of patients in each disease process, and makes individualized nutritional dietary guidance programs more targeted. Starting from the second day of the patient's hospitalization, the food eaten by the patient was weighed by professionals using the weighing method for 3 consecutive days. By recording and entering into the analysis system, it performs the calculation and analysis of food composition and nutrient intake, and analyzes it using statistical methods. The experimental results showed that patients aged 31-60 years had a higher risk of preoperative infection.

## 1. Introduction

In chronic kidney disease, with the decline of GFR and the accumulation of various metabolic wastes, patients gradually experience different degrees of loss of appetite. Urinary protein loss and a calorie-deficient diet are independent risk factors for the development of chronic kidney disease, which significantly affect prognosis. Infections not only impair organ function, but increase the complexity of treatment and the risk of patient death. It also imposes a psychological and economic burden on the patient and their family, and it is also a waste of resources for transplantation. Helping patients establish a correct health concept, apply their own knowledge and skills to implement self-management, and improve their own management level. It will help the patient's health status and quality of life to maintain a satisfactory state.

Regarding nosocomial infection, relevant scientists have done the following research. Given the clinical and economic consequences of this largely preventable injury to patient safety, the prevention of healthcare-associated infections remains an international priority. Important progress has been made in preventing nosocomial infections, but thorny issues remain. It includes how to consistently improve hand hygiene rates and further reduce device-related complications, such as catheter-related urinary tract infections. By incorporating approaches outside of traditional biomedicine, Saint may hope to provide patients with the safe care they expect and deserve [1]. The aim of the Azeredo A study was to assess the impact of ICM on the incidence of tuberculosis in healthcare workers. He conducted a retrospective records study at a comprehensive tertiary care university hospital. He reviewed all tuberculosis case reports from medical staff at the hospital. He measured TB incidence to assess the impact of implementing ICM. Tuberculosis incidence can be reduced through tuberculosis infection control programmes, surveillance, screening, training, and education [2]. Choi Y H pointed out that the novel coronavirus infectious disease pandemic poses a huge threat to medical institutions that treat patients with underlying diseases. The spread of the outbreak to hospitals must be prevented and minimized. Triage of symptomatic patients, healthcare workers, paramedics and visitors must be implemented into the entry system. To minimize outbreaks, early suspicion and detection, regular environmental cleaning and disinfection, appropriate personal protective equipment should be applied and monitored [3]. At present, the main problem of nosocomial infection is that the detection accuracy is not high.

Regarding the evaluation of economic burden, relevant scientists have done the following research. Mohd-Tahir NA aimed to systematically analyze the available evidence on health care costs associated with osteoporosis-related hip fractures in Asia. He retrieved and analyzed total costs, cost components, and length of hospital stay associated with hip fracture care. The study design was also qualitatively analyzed. There is a lack of disease research burden on osteoporosis in the Asian region. For the few available studies, methods for assessing the economic burden of disease lack standardization [4]. Wang A Y describes the symptom burden of patients diagnosed with hematological malignancies in adolescence and young adulthood, and the feasibility of incorporating palliative care into the outpatient, multidisciplinary AYA leukemia clinic at an academic medical center. Treated leukemia patients and surviving AYA patients experienced high symptom burden and low QOL. In an outpatient multidisciplinary setting, it is feasible for him to assess symptom burden and provide early palliative care focused on symptom management [5]. Leticia conducted cost comparisons and budgetary implications of mepolizumab use from a national health system perspective. Among the alternatives evaluated, inhaled systemic corticosteroids plus long-acting agonists and oral systemic corticosteroids in patients with nonimmunoglobulin-mediated severe allergic asthma, and immunoglobulin-mediated eosinophilic allergic asthma in combination with omalizumab were included [6]. J Dahham conducted a systematic literature search containing data on the prevalence or incidence-based cost of multiple sclerosis in low- and middle-income countries. Cost ratios were similar across grades of multiple sclerosis severity, making comparisons between studies by disease severity feasible. Cost drivers were primarily DMT and relapse treatment, which was consistent across studies. However, the distribution of cost components varies with disease severity [7]. The above studies conducted a detailed analysis of the application of nosocomial infection and economic burden assessment. It is undeniable that these studies have greatly promoted the development of the corresponding fields. We can learn a lot from methodology and data analysis. However, there are relatively few studies on nosocomial infection for economic burden assessment, and it is necessary to fully apply these techniques to research in this field.

By dividing the included patients into 4 groups according to the degree of disease progression, the proportion of patients' nutrition was obtained. The energy data of the four groups of patients were 1794.6, 1276.14, 1051.38 and 998.15, respectively. The proportion of protein was 14.15%, 14.96%, 15.38% and 14.92%, and the proportion of fat was 16.74%, 18.23%, 14.52% and 14.02%, respectively. The most infected patients were hospitalized for 8-15 days, reaching 145.

## 2. Method of Related Factors of Nosocomial Infection

Definition of Chronic Kidney Disease: Chronic kidney structural and functional impairment of various causes (history of kidney damage greater than 3 months). It includes normal and abnormal renal GFR pathological damage, abnormal blood or urine components, and abnormal imaging examinations, or unexplained decline in GFR (<60ml/min·1.73m^2^) for more than 3 months, which is CKD.

The diseases that cause chronic kidney disease include various primary and secondary glomerulonephritis, renal tubular damage and renal vascular lesions. Chronic kidney disease can be divided into five stages according to GFR. Early detection and early intervention can significantly reduce the complications of CKD patients and significantly improve the survival rate. For the treatment of CKD, it includes treatment of the primary disease, management of various risk factors, and delaying the progression of chronic renal insufficiency. When CKD patients progress to stage 5, renal replacement therapy should be performed promptly.

Nosocomial infections, also known as hospital-acquired infections, are infections in hospitalized patients. It includes infections acquired during hospitalization, infections acquired after discharge, and infections acquired by hospital staff while working in the hospital. It does not include infections that started before admission or that already existed at the time of admission. Surgical patients not only suffer from various invasive operations, but also suffer from blows from the operation. In addition, surgeons are worried about the complicated operation process and the long operation time. After the operation, a large number of antibiotics are used. It makes surgical patients susceptible to nosocomial infections [8].

In different stages of CKD, its clinical manifestations are also different. Before CKD stage 3, patients may have no symptoms, or only mild discomfort such as fatigue, backache, and increased nocturia. A small number of patients may have loss of appetite, metabolic acidosis and mild anemia. After CKD stage 3, the above symptoms become more obvious, and further aggravate after entering the stage of renal failure. Hypertension, heart failure, severe hyperkalemia, acid-base balance disorders, gastrointestinal symptoms, anemia, abnormal mineral bone metabolism, hyperparathyroidism, and central nervous system disorders can sometimes occur. It can even be life-threatening.

In order to do a good job in the prevention and control of nosocomial infection, it is necessary to understand the epidemiological characteristics of nosocomial infection. Nosocomial infection has three important links: the source of infection, the route of infection and the susceptible population. There are many pathogenic bacteria in nosocomial infection, mainly Gram-negative bacteria. There are many types of pathogens in hospital infection, including bacteria, fungi, rickettsia, actinomycetes, etc. With more and more pathogens infecting, many normal bacteria or opportunistic pathogens that are not easy to cause disease in the human body have become popular strains, and there are more and more types of viruses that cause nosocomial infections. There are some significant regional differences in the distribution of major pathogenic bacteria species in nosocomial infections [9].

Predisposing factors for CKD are: age (such as old age), family history of CKD (including hereditary and non-hereditary kidney disease), diabetes, hypertension, obesity-metabolic syndrome, high protein diet, hyperlipidemia, hyperuricemia autoimmune disease, urinary tract infection or systemic infection, hepatitis virus (such as hepatitis B or C virus) infection, urinary calculi, urethral obstruction, urinary or systemic tumor, history of nephrotoxic drug use, cardiovascular disease, anemia, smoking, low birth weight, etc. Other risk factors include environmental pollution, low economic level, low medical insurance level, and low education level.

There are many risk factors for nosocomial infection. Common factors include: in terms of objective conditions, patients with low autoimmunity after hospitalization, such as younger or older age, underlying diseases, malignant tumors, chronic diseases, etc. In terms of subjective conditions, invasive operations of hospital medical equipment, such as the use of ventilator intubation, central venous intubation, urinary catheter intubation, postoperative drainage tube placement, implantation of artificial materials, etc., patients use various drugs after surgery. For example, the use of antibiotics produces drug resistance, the use of glucocorticoids, etc., postoperative radiotherapy and chemotherapy drugs are used in tumor patients. In other aspects, it includes such as long postoperative hospital stay, long operation duration, etc. [10]. There are many factors that cause nosocomial infection, and different influencing factors cause different infections in different patients, but the most important thing is to do a good job in the publicity and education of nosocomial infection prevention and control knowledge. It needs to strengthen and improve the awareness of infection among medical staff, do a good job of aseptic operation in surgery, and disinfect various surgical instruments and items. At the same time, it is necessary to do a good job in hospital infection control. Especially for the monitoring and management of hospitals, by taking effective infection prevention measures, it can improve the management level of hospitals and minimize the incidence of nosocomial infections [11].

When kidney function decreases, the metabolic status of multivitamins in the body usually changes. The causes of abnormal vitamin metabolism may include: anorexia, anorexia, or insufficient vitamin content due to food intake or cooking; increased body clearance or degradation rate; increased plasma vitamin-binding protein levels.

The monitoring of nosocomial infection can be divided into comprehensive monitoring and targeted monitoring. Comprehensive surveillance refers to the comprehensive monitoring of nosocomial infections and related sources of infection among hospital staff and patients to understand epidemiological indicators, such as infection prevalence among hospital staff and patients and within sectors and the importance of different risk factors. Targeted surveillance is defined as a special type of surveillance used to focus limited human and material resources on the most important issues after a thorough understanding of nosocomial infections [12]. The main tasks of fixed-point monitoring include conducting special monitoring research on key departments, risk groups and sensitive areas in the hospital. By analyzing and investigating the risk factors associated with nosocomial infections, it predicts the occurrence of different types of nosocomial infections to improve the management of nosocomial infections related to exposure to relevant risk factors. Since it is a lifelong disease, preventing and treating kidney disease is not limited to treatment. Patients' active lifestyle changes, active participation in treatment decision-making and self-care management are critical to the success or failure of disease prevention and treatment [13].

CKD patients need to be given a low-protein diet, but must ensure adequate energy intake. The source is mainly provided by carbohydrates and fats, which can not only increase the availability of protein, increase the plasma protein concentration, but also reduce the accumulation of nitrogen-containing metabolites in the kidneys, so as to ensure normal daily physiological activities and the body's anabolic needs. It is clinically recommended that the quality of protein in the diet, especially the intake of high biological value protein, should be greater than 50%, which is conducive to correcting the negative nitrogen balance.

In order to clarify the prevention and treatment goals of CKD in different stages, it is necessary to put forward the concept of tertiary prevention. The so-called primary prevention is also called primary prevention. It refers to the timely and effective treatment of existing kidney diseases or diseases that may cause kidney damage (such as diabetes, hypertension, etc.) to prevent the occurrence of chronic renal failure (CRF). Secondary prevention refers to the timely treatment of patients with mild to moderate CRF to delay, stop or reverse the progression of chronic renal failure, and prevent the occurrence of uremia. Tertiary prevention refers to the early treatment of uremia patients. It prevents the occurrence of some serious complications of uremia and improves the survival rate and quality of life of patients.

Helping patients correctly understand their own health, apply health knowledge and skills, and improve self-care ability will help them maintain good health and quality of life. It is a health behavior designed to manage symptoms and signs of disease, reduce its impact on social functioning, mood, and relationships, and manage disease in the long-term [14]. The self-management model originated in the field of psychobehavioral therapy and was subsequently applied to health education programs for patients with chronic diseases. The aim is not to cure disease, but to enable patients to lead more independent and healthy lives through effective self-management interventions. It maintains the patient at a satisfactory level of health and function. Due to its low cost and wide coverage, this model is cost-effective and can simultaneously serve a large number of patients with different diseases, especially chronic diseases [15]. As shown in Figure 1, the application of neural network model in hospital infection.

Figure 2 shows the neural network topology, and the related algorithms of the neural network are as follows.


(1) $$\begin{array}{c} Z_{k}=f\left(\sum_{u=1}^{b}y_{ku}m_{u}+j_{k}\right), \end{array}$$

(2) $$\begin{array}{c} D_{v}=f\left(\sum_{u=1}^{w}q_{ku}Z_{k}+s_{v}\right). \end{array}$$

*w*- the number of nodes in the hidden layer

*b*- the number of nodes in the input layer

(3) $$\begin{array}{c} E_{y}=\begin{array}{c} 1\\ 2 \end{array}{\sum_{v=1}^{a}\left(t_{v}^{y}-n_{v}^{y}\right)}^{2}, \end{array}$$

(4) $$\begin{array}{c} E=\begin{array}{c} 1\\ 2 \end{array}{\sum_{y=1}^{l}\sum_{v=1}^{a}\left(t_{v}^{y}-n_{v}^{y}\right)}^{2}. \end{array}$$

*l*- Number of samples

*t*_*v*_^*y*^- Expected output

(5) $$\begin{array}{c} \Delta q_{vk}=-\mu \begin{array}{c} \partial E\\ \partial q_{{}_{vk}} \end{array}. \end{array}$$

*μ*- Learning rate

(6) $$\begin{array}{c} \Delta q_{vk}=\sum_{y=1}^{l}\sum_{v=1}^{a}\mu f^{\prime }\left(D_{v}\right)\cdot Z_{k}, \end{array}$$

(7) $$\begin{array}{c} \Delta y_{ku}=\sum_{y=1}^{l}\left(-\mu \begin{array}{c} \partial E\\ \partial y_{ku} \end{array}\right). \end{array}$$

Δ*q*_*vk*_- The weights of each neuron in the output layer

Δ*y*_*ku*_- Hidden layer weights

(8) $$\begin{array}{c} \gamma_{zk}=-\begin{array}{c} \partial E_{y}\\ \partial Z_{k} \end{array}\cdot \begin{array}{c} \partial Z_{k}\\ \partial D_{k} \end{array}. \end{array}$$

*γ*_*zk*_- Error signal

(9) $$\begin{array}{c} \tau \left(m\right)=\begin{array}{c} 1\\ 1+e^{-im} \end{array}. \end{array}$$

*τ*(*m*)- Nonlinear activation function

(10) $$\begin{array}{c} T=T_{0}+\begin{array}{c} \alpha \\ 2b \end{array}\sum_{q}q^{2}, \end{array}$$

(11) $$\begin{array}{c} q=q-\mu \begin{array}{c} \partial T_{0}\\ \partial q \end{array}-\mu \begin{array}{c} \alpha \\ b \end{array}q. \end{array}$$

*T*_0_- Original cost function

*α*- regularization coefficient

(12) $$\begin{array}{c} q=\left(1-\begin{array}{c} \mu \alpha \\ b \end{array}\right)q-\begin{array}{c} \mu \\ a \end{array}\sum_{m}\begin{array}{c} \partial T_{m}\\ \partial q \end{array}, \end{array}$$

(13) $$\begin{array}{c} j=j-\begin{array}{c} \mu \\ a \end{array}\sum_{m}\begin{array}{c} \partial T_{m}\\ \partial j \end{array}. \end{array}$$

*q*- Weight

*j*- Threshold

(14) $$\begin{array}{c} n=F\left(m,\left\{Q_{u}\right\}\right)+m, \end{array}$$

(15) $$\begin{array}{c} \begin{array}{c} \partial n_{v}\\ \partial Z_{k} \end{array}=f^{\prime }\left(D_{v}\right)q_{vk}. \end{array}$$

*m*- input vector

*n*- output vector

The theoretical foundations of self-management are social cognitive theory, self-efficacy theory and self-determination theory. Self-management theory is a new model of chronic disease management in which health professionals collaborate with patients. By teaching them basic health knowledge and skills, it enables them to manage and control their disease through health education. It consists of three main elements: daily life management, medical disease management, and cognitive emotion management. Self-management is a sociological indicator of quality of life, state, behavior, and attitude, so its measurement must be based on sociological scales [16].

Self-management education is a better way to improve patients' self-management abilities, which has been demonstrated in other chronic diseases such as hypertension and diabetes. In addition to improving patients' self-management skills, as well as their behavior and self-efficacy, it reduces emergency room visits, reduces stress and burden on hospitals, delays or preventable complications, and improves patients' overall health and quality of life . As the patient's disease progresses and lifestyle changes, the patient's inability to adapt to these changes, and the long-term effects of the disease limit physical activity, forcing people to adopt a less active lifestyle. These may be the main reasons for the decline in physical activity levels [17]. This suggests that changing and improving patient self-care behaviors by treating thousands of premature babies is not only possible in theory, but also effective in practice. Reports suggest that self-care education improves patient self-care and leads to the development of health-promoting behaviors [18].

Individuals are directly responsible for maintaining their own health, and maintaining health is largely dependent on their own efforts. Individuals are fully capable of maintaining their own health, coping with illness and recovering. Kidney disease is a slow and long-term disease process, and its effective treatment cannot be solved by drugs alone. It also needs to be combined with holistic interventions such as dietary changes, appropriate physical activity, and regular monitoring of renal function [19]. These interventions are delivered through patient self-management behaviors, whereby patients spend less time under the direct supervision of health professionals and more time in community and family life, known as self-management time. Therefore, good self-management is critical to the long-term survival and quality of life of patients. Studies have shown that self-care programs not only improve patient quality of life, but also increase self-efficacy and adherence to care, and reduce hospital admissions and emergency care [20].

While the focus is on patient self-care, family support is an important element of social support. It has a large impact on the patient's self-care behavior, and it is important to promote the development of a family support system and establish close cooperation between family members. In addition to supporting, monitoring, and supervising the patient's diet, family members can comfort the patient, reduce emotional distress, and relieve tension and anxiety. However, at present, the involvement of family members in the management of the disease is limited for several reasons [21]. Through comprehensive health education, patients and their families can fully understand the disease, view the disease from a scientific perspective, and gain the knowledge and skills to manage their own health. This motivates patients and their families to fully participate in health self-management models, develop their skills in this area, and enable patients to have a good quality of life [22].

The dietary habits of patients with kidney disease are closely related to health status, quality of life, survival rate, and complications such as hyperkalemia, renal bone disease, and hypertension. Therefore, dietary management is the most important and basic self-management measure. Therefore, patients should be actively encouraged to change their dietary habits and choose a diet that is low in protein, high in calories and vitamins, low in and potassium, and moderate in water and salt [23]. Soy protein is a special case when it comes to limiting plant protein intake. Research and clinical observations have shown that a soy protein diet can not only reduce proteinuria and improve nutritional status, but also protect kidney function and delay the development of chronic kidney disease. It should also advise patients to avoid spicy foods such as chili, mustard, and pepper, reduce the intake of fried and cold foods, and pay attention to dietary hygiene [24].

Moderate physical activity can improve hypertension, anemia and malnutrition. It increases the body's resistance and improves the patient's physical and mental health. It can also help control blood sugar levels in people with diabetes and slow the progression of the disease. Therefore, it should encourage patients to adjust the time, content and amount of work or housework according to their current physical condition and ensure a regular lifestyle. It should encourage the patient to establish an appropriate exercise and rest program. Exercise programs should include aerobic, endurance, and range-of-motion exercises, starting with low-intensity exercises such as walking and tai chi and following a gradual increase to avoid fatigue [25].

Nutritional status is very important for patients with kidney disease to maintain good health, and various nutrient metabolism disorders are one of the main clinical manifestations. Studies have shown that PEM can be one of the independent factors affecting kidney disease. Patients with poor nutritional status have longer hospital stays, higher costs and are more prone to complications. Good nutritional status can improve patients' immunity and reduce clinical symptoms. Nutritional therapy can maintain the patient's normal nutritional needs and correct the imbalance of amino acids and electrolytes in the body. It is in positive nitrogen balance or close to it. This can improve the patient's disease resistance, lead to remission, and prolong life expectancy. The patient's appetite is greatly affected by the disease, which will greatly affect the intake and absorption of nutrients, which is detrimental to the disease [26].

In terms of payments, this “single bill“ approach could lead to more people tending to be admitted to the hospital. Factors affecting hospitalization costs were: length of hospital stay, average number of hospitalizations, number of more than four hospitalizations, level of hospitalization, age group, gender, occupational status, and contagiousness of the disease. Hospitalization was the determining factor. The number of days in hospital, the quota of more than 4 days, the level of hospitalization, age group, gender, occupational status, and contagiousness of the disease were considered objective factors for the patient or disease, while the average hospitalization rate was a subjective human factor. Hospitals with different rates may have different costs for treating the same disease, and the insured and the hospital may not receive the same comprehensive payment amount.

The current major medical insurance system adopts a single total billing model, and the main billing method for medical insurance is the average bill per unit of service. Except for the hospital level, there is a high correlation between the hospital's previous payment level and the hospital's payment rate, but there is no quantitative standard for determining the hospital's payment rate. Hospitals and individuals pay different costs between hospitals at different levels of the same disease and between hospitals within a level. Because payment standards directly affect a hospital's reimbursement levels and financial returns, it affects how a hospital treats insured patients. By playing a game with the government, hospitals can reduce the number of treatments to make a profit, or they can deliberately violate quotas so that they can be adjusted the following year.

The cost of hospital care depends largely on the type and severity of the disease. Factors affecting hospital care costs are related to the patient's situation and social characteristics, but also to the patient's ability to pay and how the cost is paid. The medical insurance management department has introduced a relatively strict hospital fee fixing system, which has slowed down the growth of hospital fees to a certain extent. Areas B and C implement relatively loose medical insurance control policies, which results in higher per capita medical insurance patients in areas B and C than those in the city. On the other hand, government-funded medical services implement a project approval and comprehensive control system, and implement a stricter cost control and cost sharing system. This shows that the cost-sharing policy has a direct impact on the hospitalization expenses of patients, and the implementation of a fixed payment system and strict control of medical insurance cost-sharing. It can force the medical behavior of medical institutions and medical personnel, and control the cost of treatment. The economic burden evaluation process is shown in Figure 3.

Equity in the financing and coordination of Medicare benefits should be further promoted. The scope of coordinated payments should be expanded, for example, by specifying a certain percentage of payments for general outpatient clinics and increasing the percentage of payments. The flat rate of hospitalization is the most important determinant of the hospitalization cost of medical insurance, and the flat rate of hospital is basically a method of per capita payment. However, the uniform charges of hospitals vary from medical institution to medical institution, and there is no objective standard, which is absurd. After comparing the hospital expenses of insured and uninsured hospitals in different regions, it is found that the per capita hospital expenses of patients in different regions vary greatly, and there are also differences within the same hospital. This suggests that payment systems and affordability can influence physicians' treatment behaviors, and thus health care costs. A reasonably strict health insurance policy can help keep costs in check.

Medical insurance acts as a “reservoir and stabilizer“ in maintaining social stability, whether the insurance fund can break even. This is an issue of great concern to the medical insurance administration. By using historical data and appropriate forecasting methods to accurately predict the expenditure of medical insurance funds, it is conducive to the further adjustment and improvement of medical insurance policies. The advantage of multiple linear regression analysis is the ability to analyze the determinants of health care costs, but it cannot identify dynamic trends over time in the population studied. Dynamic grey models do not have strict requirements on sample size and probability distribution. It is suitable for predicting relatively stable short-term trends, but it is not effective for predicting cyclically changing time series. Although a neural network model can theoretically approximate rational functions with arbitrary accuracy, it requires more relevant data. The definition of network levels and nodes needs to be learned repeatedly. The modeling process often encounters local minima. The selection of network levels and nodes also needs to be checked repeatedly, which is difficult to implement. As shown in Figure 4, the medical expenses are shown.

The financial burden of disease refers to the economic loss to patients and society, including financial resources used to prevent and cure serious illness, disability, and premature death. The financial burden of disease is divided into direct and indirect financial burdens. The direct economic burden of a disease is the total annual cost of preventing and treating the disease, including various social and family costs directly related to the treatment, diagnosis, treatment and rehabilitation of the disease. One of the components is related to the cost of purchasing medical services. Direct medical expenses include outpatient treatment, inpatient treatment, and drug costs. It includes over-the-counter ingredients, rehabilitation costs, and other medical expenses. The second part refers to the cost of obtaining medical services, including direct non-medical expenses such as transportation, meals, accommodation, escort services, etc. The indirect economic burden of illness is the loss of current and future social and family value due to lost work time or reduced ability to work due to illness, disability or death.

## 3. Experiments for Related Factors of Nosocomial Infection

The patients to be included will be divided into 4 groups according to the degree of disease progression.  Table 1 shows the proportion of nutrition in patients. There was no significant difference between groups in the proportion of each group, and energy intake decreased from CKD stage 3.

Table 2 shows a comparison of the general data of the patients. It can be seen that there are very many patients over the age of 50 and fewer patients under the age of 31.

The overall self-management status of the patients was investigated.  Table 3 shows the survey results, and Table 4 shows the preoperative status of the recipients. The scores of each dimension from high to low were treatment management, diet management and physical activity management.

The patient's surgical status is shown in Figure 5. It can be seen from the figure that the operation type of kidney transplant recipients is mainly emergency.

The shortest postoperative infection time was 5 days, the longest was 2675 days, and the median was 92 days. As shown in Figure 6, the infection rates at different time periods after surgery are shown.

As shown in Figure 7, the postoperative infection rates of patients in different age groups are shown. It can be seen that the proportion of people aged 31-60 years old is higher, and preoperative infection is generally higher than postoperative infection

The incidence of postoperative infection was higher in all groups, suggesting that nosocomial infection control measures should be strengthened to reduce the incidence of infection in patients with longer postoperative hospital stays. Because some patients were not hospitalized after infection, or were not treated at the hospital where the infection was investigated, it is possible that it underestimated the number of outpatient infections. The hospital strictly complied with infection control requirements for cleaning and disinfection during hospitalization, and the reason for the high infection rate after discharge needs further investigation. Patients who have been in the intensive care unit for a long time after surgery should have a drug susceptibility test immediately, and sensitive drugs should be selected according to the results of the drug susceptibility test. Renal disease patients are a high-risk group for postoperative infection, not only have a high incidence of infection, but also have a high mortality rate due to infection, and patients are prone to multiple infections.

By incorporating patients into the management of chronic disease patients in the community, as key control objects, health records are established, infection risk factors are intervened, and regular follow-up visits are performed. Through the introduction of relevant policies, it provides medical subsidies to patients. It incorporates commonly used drugs after surgery into the scope of medical insurance reimbursement to reduce the financial burden of patients.

Calcium is an important component of the human body, and some serious complications in CKD patients are caused by abnormal calcium and phosphorus metabolism. The pathogenesis may be due to decreased urinary excretion of phosphorus in the early stages of GFR reduction. The accumulation in the body increases, the blood calcium decreases, and the body's regulating system is to maintain the normal blood calcium and blood phosphorus. It causes a compensatory increase in the secretion of parathyroid hormone to maintain a balanced state by smoothing the excretion of phosphorus from the kidneys.

## 4. Conclusion

Switching to renal replacement therapy is an end point for only a minority of patients. People with chronic kidney disease had significantly shorter life expectancies than controls of the same age. One of the important reasons is the premature death of patients with chronic kidney disease due to combined cardiovascular and cerebrovascular diseases. In addition, due to the influence of physical, economic, social, family and other factors, patients usually face severe psychological pressure and show fear of disease. Patients lack confidence in treatment, poor compliance, and even suicidal tendencies. This study analyzed the related factors of nosocomial infection in patients with chronic kidney disease. Postoperative hospital stay and community infection should be paid attention to. Given the limitations of manpower, time, etc., this study adopted a cross-sectional design and failed to observe the long-term effect of the project intervention, which may affect the inference of the results.

## Figures and Tables

**Figure 1:** Application of Neural Network Model in Nosocomial Infection.

**Figure 2:** Neural Network Topology.

**Figure 3:** Economic Burden Evaluation Process.

**Figure 4:** Medical expenses.

**Figure 5:** Patient's surgical status.

**Figure 6:** Infection rates at different time periods after surgery.

**Figure 7:** Postoperative infection rate in patients of different age groups.

**Table 1:** The proportion of nutrition in patients.

Index	Grouping			
	CKD2	CKD3	CKD4	CKD5
Energy (kcal)	1794.6	1276.14	1051.38	998.15
Protein (%)	14.15	14.96	15.38	14.92
Fat (%)	16.74	18.23	14.52	14.02

**Table 2:** Comparison of patient general data.

Age	Intervention group		Control group	
	Quantity	Percentage	Quantity	Percentage
<31	4	8.3	3	6.2
31-50	10	20.8	19	39.6
>50	34	70.8	25	54.2

**Table 3:** Rank Distribution of Self-Management Score Indicators.

Project	Good		Medium		Bad	
	Number of cases	Percentage (%)	Number of cases	Percentage (%)	Number of cases	Percentage (%)
Treatment management	11	11.5	65	68.8	20	19.8
Diet management	10	10.4	61	63.5	25	26.03
Physical activity management	9	9.4	59	60.5	28	30.2

**Table 4:** Recipient's preoperative condition.

Variable	Grouping	Number of people	Composition ratio
PRA	Negative	339	99.1
	Positive	4	0.9

Dialysis before surgery	Yes	304	88.9
	No	39	11.1

## Data Availability

No data were used to support this study.
